The article "Sanguinarine-Chelerythrine Fraction of Coptis chinensis Exerts Anti-inflammatory Activity in Carrageenan Paw Oedema Test in Rats and Reveals Reduced Gastrotoxicity" was published in 2022. Journal: Oxid Med Cell Longev.

# Sanguinarine-Chelerythrine Fraction of *Coptis chinensis* Exerts Anti-inflammatory Activity in Carrageenan Paw Oedema Test in Rats and Reveals Reduced Gastrotoxicity

**DOI:** 10.1155/2022/1504929

**Published:** 2022-03-16

**Authors:** Maciej Danielewski, Sylwia Zielińska, Agnieszka Matuszewska, Wojciech Słupski, Maciej Włodarczyk, Izabela Jęśkowiak, Benita Wiatrak, Krzysztof Kowalski, Anna Jezierska-Domaradzka, Piotr Ziółkowski, Adam Szeląg, Beata Nowak

**Affiliations:** ^1^Department of Pharmacology, Wroclaw Medical University, J. Mikulicza-Radeckiego 2, 50-345 Wrocław, Poland; ^2^Department of Pharmaceutical Biotechnology, Wroclaw Medical University, Borowska 211, 50-556 Wrocław, Poland; ^3^Department of Pharmacognosy and Herbal Medicines, Wroclaw Medical University, Borowska 211A, 50-556 Wrocław, Poland; ^4^Department of Pathology, Wroclaw Medical University, K. Marcinkowskiego 1, 50-368 Wrocław, Poland

## Abstract

Inflammatory diseases are a common therapeutic problem and nonsteroidal anti-inflammatory drugs are not deprived of side effects, of which ulcerogenic activity is one of the most frequent. The aim of the study was to evaluate the anti-inflammatory activity of the sanguinarine-chelerythrine (SC) fraction of *Coptis chinensis* and its influence on the integrity of gastric mucosa. The study was conducted on sixty male rats randomly divided into six experimental groups: two control groups (a negative control group CON and a positive control group CAR); three groups receiving an investigational fraction of *C. chinensis* (1, 5, 10 mg/kg *i.g.*) named SC_1_, SC_5_, and SC_10_, respectively; and a group receiving indomethacin (IND) (10 mg/kg *i.g.*) as a reference drug. In all animals, the carrageenan-induced paw oedema was measured; PGE_2_ release, TNF*α* production, and MMP-9 concentration in inflamed tissue were determined. Additionally, the macroscopic and microscopic damage of gastric mucosa was evaluated. Administration of SC dose-dependently inhibited the second phase of carrageenan rat paw oedema and PGE_2_ release, decreased the production of TNF*α*, and reduced the concentration of MMP-9, and the efficacy of the highest dose was comparable to the effect of IND. Contrary to IND, no gastrotoxic activity of SC was detected. The investigated sanguinarine-chelerythrine fraction of *C. chinensis* seems to be a promising candidate for further research on new anti-inflammatory and analgesic drugs characterized with a safer gastric profile compared to existing NSAIDs.

## 1. Introduction

Inflammation is an important defence mechanism protecting the organism against harmful stimuli, such as bacteria, viruses, and fungi. However, excessive inflammation is involved in the development of multiple diseases, e.g., destructive arthritis, inflammatory colitis, atherosclerosis, and diabetes mellitus. Chronic inflammatory diseases belong to the main problems affecting the lifestyle and quality of life of millions of people all over the world. However, existing therapies are not always effective and they are often associated with the burden of adverse effects that limit their usage. Nonsteroidal anti-inflammatory drugs (NSAIDs) are very efficient and widely used in the treatment of various inflammatory conditions, but gastrointestinal complications frequently constrict their application. In this context, there is a great need to look for new agents that, on one hand, would be effective in the management of pain and inflammation and, on the other hand, would be safer than existing ones. Natural compounds with anti-inflammatory activity are a large and important group of pharmaceuticals that might be used in the treatment of various inflammatory diseases.

Inflammatory stimuli (e.g. foreign organisms, tissue damage, or antigens) activate an immune response that under some conditions may be deleterious for the host and lead to chronic inflammation. The cell damage associated with inflammation acts on the cell membrane to release leukocyte lysosomal enzymes that liberate among others arachidonic acid (AA). Mobilized AA is then converted into a variety of prostanoids by means of cyclooxygenases 1 and 2 (COX-1 and COX-2). Prostaglandin E_2_ (PGE_2_) and prostacyclin (PGI_2_) are predominant prostanoids involved in inflammatory reactions. They enhance oedema by increasing vascular permeability and promoting leukocyte infiltration. They may regulate lymphocyte function, and PGE_2_ with thromboxane A_2_ (TXA_2_) plays an important role in T-lymphocyte development. However, prostanoids are not only involved in the pathological process associated with inflammation. They are also engaged in keeping homeostasis; e.g., in the gastrointestinal tract, the integrity of gastric mucosal defence relies on the continuous synthesis of prostanoids.

*Coptis chinensis*, with its broad bioactive potential, is one of the 50 most important herbs in traditional Chinese medicine (TCM) [1]. TCM it has been used to treat various inflammatory diseases, high fever, toothache, gastrointestinal disorders, diabetes, and skin diseases for thousands of years [2]. Various contemporary studies confirmed the anti-inflammatory activity of *C. chinensis* [3–6]. However, they attributed the anti-inflammatory properties of the investigated extract mainly to the activity of berberine, which is the most abundant alkaloid found in *C. chinensis*.

Sanguinarine and chelerythrine (Figure 1) are benzophenanthridine alkaloids widely distributed in plants belonging to the *Papaveraceae, Fumariaceae*, *Rutaceae*, *Ranunculaceae*, and *Meliaceae* families. Apart from *C. chinensis*, these substances were also found as one of the most abundant compounds in *Chelidonium majus* L. (CM) [2, 7–10]. Both alkaloids were also detected in other plant species, such as *Sanguinaria canadensis*, a North American plant used as a dental antibacterial agent and as an antiarthritic and anticancer treatment [11].

Sanguinarine is a promising pharmacologically active substance of plant origin, because so far, in addition to its anti-inflammatory effect, its potential therapeutic use, e.g., in the treatment of osteoporosis (F. [12]), hypertension [13, 14], heart failure [15], atherosclerosis [16], cancer [17], infectious diseases (Q. [18, 19]), or asthma [20], has been reported. Very similar results were obtained with chelerythrine (H. [21]; N. [22–26]). Taking into account a considerable amount of reports confirming the positive effect of both alkaloids on various pathologies, the knowledge about the anti-inflammatory activity and possible use of these compounds in the treatment of inflammatory diseases should also be constantly expanded.

Zielińska et al. [27] reported that chelerythrine decreased the TNF*α* secretion in human neutrophils and sanguinarine was the most potent inhibitor of IL-1*β* secretion among CM alkaloids. Other authors informed that anti-inflammatory activity of sanguinarine and chelerythrine may be a consequence of their inhibitory influence on the secretion of CCL-2, IL-6, and IL-1 RA [28]. Sanguinarine was also reported to be a potent inhibitor of the TLR4/NF*κ*B signal transduction [4].

The above promising reports prompted us to examine the potency and therapeutic application of these two alkaloids isolated from *C. chinensis.* The aim of the study was to investigate the anti-inflammatory properties of sanguinarine-chelerythrine fraction isolated from *C. chinensis* and its influence on the integrity of gastric mucosa.

## 2. Materials and Methods

### 2.1. Chemicals and Materials

The following drugs and chemicals were used to perform the experiment: carrageenan (Sigma-Aldrich, Steinheim, Germany) and indomethacin (Sigma-Aldrich, Steinheim, Germany); 0.9% saline solution (Polpharma, Starogard Gdanski, Poland); ketamine and xylazine 20 mg/mL (Sedazin®, Biowet, Pulawy, Poland); ketamine 100 mg/mL (Biowet, Pulawy, Poland); and formalin 37% sol (Chempur, Piekary Slaskie, Poland). Other used chemicals were included in the commercially available kits.

### 2.2. Plant Compound Preparation

Sanguinarine-chelerythrine fraction of *C. chinensis* extract was used in the carrageenan paw oedema test in rats. The fraction containing both alkaloids was isolated as a mixture (0.2 : 1 *w*/*w*) from *C. chinensis rhizoma* (19 g/100 g yield) as described previously [10].

### 2.3. Animals

The study was conducted on sixty male Wistar rats (weighing 224.7 ± 10.0 g) purchased from the Animal Research Centre at Wroclaw Medical University (Wroclaw, Poland). Rats were housed in pairs in transparent polypropylene cages, under standard conditions of temperature (21-23°C), humidity (60–70%), and a light-dark cycle (12 : 12 h). Animals were fed a standard rodent diet (LSM, Agropol, Motycz, Poland), with access to food and water was *ad libitum*.

### 2.4. Ethics Statement

The study protocol was approved by the First Local Ethics Committee for Animal Experiments in Wroclaw, Poland. All animal experiments were performed in accordance with ARRIVE guidelines and the EU Directive 2010/63/EU for animal experiments.

### 2.5. Drug Administration

Acclimated animals were randomized into six experimental groups of ten animals each: two control groups (a negative control group (CON) and a positive control group (CAR)) receiving 0.9% saline solution intragastrically (*i.g.*) (3 mL/kg), three groups receiving investigational fraction of *C. chinensis* containing sanguinarine and chelerythrine (1, 5, and 10 mg/kg *i.g.* in saline solution 3 mL/kg) named SC_1_, SC_5_, and SC_10_, respectively, and a group receiving indomethacin (IND) (10 mg/kg *i.g.* in saline solution 3 mL/kg) as a reference drug.

### 2.6. Carrageenan Paw Oedema Test

One hour after administration of the appropriate experimental substance, a single injection under the plantar aponeurosis of the right hint footpad was performed. Animals received either 100 *μ*L of 0.9% saline solution (CON group) or 100 *μ*L of 1% carrageenan solution (all other groups) as described by other authors [29, 30] [29, 30]. The paw volume was measured with a plethysmometer (Plethysmometer 37140 Ugo Basile, Gemonio, Italy) five times in each animal: before the injection of carrageenan/saline solution and 1, 2, 3, and 6 hours after the injection. After the last measurement, under deep anaesthesia with ketamine (60 mg/kg, *i.p.*) and xylazine (10 mg/kg, *i.p.*), rats were euthanized by dislocation of cervical vertebrae C6-C7.

Paw oedema in the individual animal was defined as a change of its paw volume:

(1) $$\begin{array}{c} \text{Paw oedema}=\text{paw volume at the analyzed time point}–\text{initial paw volume}. \end{array}$$

The percentage of the inhibition of the inflammatory reaction was calculated with the following formula:

(2) $$\begin{array}{c} \%\text{of inhibition}=\left(1–\frac{\text{change of paw volume in the analyzed animal}}{\text{mean change of the paw volume in CAR group}}\right)\times 100\%. \end{array}$$

### 2.7. Isolation of Right Hint Paw

After euthanasia, the right hint paws were immediately cut off. The subplantar tissue was isolated and homogenized, and the obtained supernatant was frozen for further enzyme-linked immunosorbent assay (ELISA). The concentration of tumour necrosis factor alpha (TNF*α*), prostaglandin E_2_ (PGE_2_), and matrix metalloproteinase 9 (MMP-9) in the supernatant was assessed with commercial ELISA Kits (Nori Rat TNF Alfa ELISA Kit, Genorise Scientific Inc., Glen Mills, USA; Nori Rat PGE 2 ELISA Kit, Genorise Scientific Inc., Glen Mills, USA; and Nori Rat MMP-9 ELISA Kit, Genorise Scientific Inc., Glen Mills, USA, respectively) according to the manufacturer's instructions.

### 2.8. Isolation of Stomach and Collection of Gastric Juice

After euthanasia, the abdomen was opened and the stomach excised. The removed stomach was opened along greater curvature, and gastric content was rinsed with 5 mL of distilled water into a centrifuge tube. The obtained solution was centrifuged at 3000 rpm for 15 min. The supernatant was used for pH measurement. The cleaned stomach was preserved in 0.1 M phosphate-buffered saline (1 : 4 (*w*/*v*), pH 7.4) prior to macroscopic examination. Then, the stomach was fixed in 4% buffered formalin, embedded in paraffin, and cut into 4 *μ*m thick slices, which were mounted on the glass slides and stained by the routine hematoxylin-eosin (H&E) method.

### 2.9. Measurement of the pH of Gastric Juice

The pH of gastric juice was measured with GLP 21 pH meter (Crison Instruments SA, Barcelona, Spain) according to the manufacturer's instruction.

### 2.10. Macro- and Microscopic Examination of Gastric Mucosa

The damage of the gastric mucosa was assessed in macro- and microscopic examination. The severity of macroscopically visible changes in the mucous membrane was evaluated using the J-scoring method, classifying the erosions as follows: no erosions = 0; 0-1 mm in diameter = 1; 1-2 mm = 2; and greater than 2 mm in diameter = 3. The sum of these measured areas in each animal was described as the gastric index [31].

Histopathological changes of all stomach specimens were examined in a blinded way by the experienced pathologist. The inflammation process and the damage of gastric mucosa were assessed independently. The severity of the inflammation was assessed using 0-3 scale (0: no inflammation, 1: mild inflammation, 2: moderate, and 3: severe inflammation). The severity of the damage of gastric mucosa was assessed using 0-3 scale (0: no damage, 1: superficial erosion, 2: submucous ulceration, and 3: ulceration in muscularis propria). The cumulative microscopic gastric index was defined as the sum of the inflammation and damage score.

### 2.11. Statistical Analysis

All experimental data are presented as the mean values ± standard deviation (SD). Statistical differences between studied parameters were analyzed using one-way analysis of variance (ANOVA) and NIR Fischer post hoc test. The comparison of the anti-inflammatory activity of the investigated doses of the tested fraction and indomethacin was performed with the multicriteria decision analysis (MCDA) using the weighted sum model (WSM). The weights were selected based on the meaning of each bioassay. The weights were set at 0.4 for the carrageenan paw oedema test and 0.2 for the assessment of PGE_2_, MMP-9, and TNF*α* levels. All statistical analyses were performed with Statistica v. 13.1 (Tibco Software, Palo Alto, USA) with statistical significance set at *p* value < 0.05.

## 3. Results

### 3.1. Carrageenan Paw Oedema Test

Paw oedema in the experimental groups is shown in Figures 2 and 3. A significant increase in paw volume was observed in all groups that received subplantar injection of 1% carrageenan solution compared to the CON group 2 hours after the injection and sustained increase throughout the experiment. The enhancement in paw volume was lower in rats receiving indomethacin and the investigational fraction of alkaloids in both higher doses (5 mg/kg and 10 mg/kg) compared to an untreated positive control (CAR). The inhibitory effect of the lower dose (5 mg/kg) lasted shorter than the effect of the higher dose (10 mg/kg) of alkaloid fraction and indomethacin. The inhibition of the inflammatory reaction with indomethacin and the investigational fraction is presented in Figure 4. At the end of the experiment, the inhibitory effect of the highest dose of alkaloid fraction (10 mg/kg) did not differ significantly from the effect of indomethacin. Lower doses of the investigational fraction containing sanguinarine and chelerythrine (1 mg/kg and 5 mg/kg) inhibited the paw oedema to a lesser extent than indomethacin.

### 3.2. Assessment of TNF*α*, PGE_2_, and MMP-9

The enzyme-linked immunosorbent assay (ELISA) was used to assess the concentration of TNF *α*, PGE_2_, and MMP-9 in the homogenized subplantar tissue (Table 1). The injection of 1% carrageenan solution induced a potent production of TNF *α*, PGE_2_, and MMP-9, which was significantly inhibited with indomethacin 10 mg/kg and an investigational fraction of alkaloids in all examined doses (1, 5, and 10 mg/kg).

### 3.3. Histopathological Assessment of Gastric Mucosa

To assess the gastric safety profile of the investigated compounds, macroscopic (Figure 5) and microscopic (Figure 6) examinations of the stomachs were performed. The presence and severity of macroscopically visible lesions (petechiae, hemorrhagic erosions) were scored as the indicators of ulcerogenic activity (cumulative macroscopic gastric index calculated as the sum of the measured pathological areas evaluated using the J-scoring method). Macroscopic examination of the gastric mucosa demonstrated that investigational fraction of *C. chinensis* in all assessed doses caused negligible mucosal lesions (Figures 5(a)–5(c) and Table 2, *p* > 0.05*vs.* CON), whereas indomethacin given in the dose of 10 mg/kg caused significant gastric injuries (Figure 5(d) and Table 2, *p* < 0.0001*vs.* CON). The microscopic assessment was in line with the values obtained macroscopically. The stomach tissue of rats pretreated with SC fraction as well as the control rats showed no significant histopathological changes (Figures 6(a)–6(c), 6(e), and 6(f) and Table 2). The examination of stomach tissue of indomethacin-treated animals revealed inflammation and ulceration in the mucosa, confirming the ulcerogenic activity of indomethacin (Figure 6(d) and Table 2).

### 3.4. pH of Gastric Juice

A significant increase in pH of gastric juice was observed only in animals receiving a low dose (1 mg/kg) of investigational alkaloid fraction of *C. chinensis* containing sanguinarine and chelerythrine (Table 3).

### 3.5. Multicriteria Decision Analysis (MCDA)

The results obtained in the carrageenan paw oedema test and ELISA performed for three doses of investigational alkaloid fraction and indomethacin were analyzed with MCDA to compare their anti-inflammatory activity. The results of MCDA (Figure 7) showed that the investigational fraction of *C. chinensis* acted dose-dependently and it exerted a relevantly lower anti-inflammatory effect than indomethacin 10 mg/kg only if given in the lowest dose of 1 mg/kg.

## 4. Discussion

The protective effect of sanguinarine-chelerythrine fraction of *C. chinensis* on acute inflammation in rat paw was investigated in the reported study. The study showed that the investigational fraction of *C. chinensis*, especially at the highest dose of 10 mg/kg, was capable of ameliorating carrageenan-induced rat paw oedema. Additionally, it reduced the carrageenan-induced secretion of PGE_2_, TNF*α*, and MMP-9 in the rat paw. The anti-inflammatory effect of the investigational fraction of *C. chinensis* was not associated with damage of gastric mucosa. To our knowledge, this was the first study to assess the anti-inflammatory potency as well as to compare the effects of the SC fraction to the use of indomethacin in an acute inflammatory model.

One of the most commonly used tests to investigate the anti-inflammatory activity of experimental substances is the carrageenan rat paw oedema test. According to the guidelines, it is the first *in vivo* study, which should be performed after the *in vitro* tests of potentially anti-inflammatoryplant-derived substances [32]. The carrageenan exerts a biphasic inflammatory effect. The first phase lasts 1 to 2.5 hours and is associated with the secretion of histamine and serotonin at the beginning followed by kinin release. In the second phase, lasting from 2.5 to 6 h, the inflammatory reaction is mediated mainly by excessive production of PGE_2_ [33]. We observed significant paw oedema in the carrageenan-injected animals. The pretreatment with the alkaloid fraction of *C. chinensis* containing sanguinarine and chelerythrine dose-dependently inhibited the second phase of carrageenan rat paw oedema in regard to the positive control group, suggesting the inhibition of PGE_2_ release. Similar results were reported for the nonprotein fraction of *C. majus* extract that contains among others sanguinarine and chelerythrine [34] [34] [34]. In the reported study, six hours after carrageen-administration, there was no significant difference in the inhibition of the paw oedema between the animals pretreated with indomethacin (the reference nonsteroidal anti-inflammatory drug) at the dose of 10 mg/kg and those that received the highest dose of the SC fraction (10 mg/kg). However, lower doses of an investigational fraction of *C. chinensis* were less potent than the reference drug.

In the present study, we found a significant increase in the levels of inflammatory mediators such as PGE_2_ and TNF*α* in the paw of carrageenan-administered animals. Prostaglandin E_2_ is the most abundantly detected PG in various tissues and exerts versatile physiological and pathological actions via four EP1–4 receptor subtypes [35]. The role of PGE_2_ in acute inflammation was initially associated with vasodilatation of vascular smooth muscle cells via the EP2/EP4 receptors; then, it was demonstrated that PGE_2_ induces mast cell activation via EP3 and consequently enhances vascular permeability, contributing to PGE-induced acute inflammation [36]. Moreover, PGE_2_ promotes T_h_1-cell differentiation, T_h_17-cell proliferation, and production of proinflammatory IL-22 from T_h_22 cells *in vitro* via EP2 and EP4 and intensifies chronic inflammation mostly via the EP4 receptor [35]. In turn, TNF*α* is believed to be a key proinflammatory cytokine involved in many pathological processes. TNF*α* among others can stimulate the overexpression of COX-2 and subsequently the overproduction of PGE_2_ [37]. The pretreatment with the alkaloid fraction of *C. chinensis* containing sanguinarine and chelerythrine (in all investigated doses) decreased the level of PGE_2_ in the paw after the carrageenan injection. This observation supports the hypothesis about the inhibition of PGE_2_ synthesis, which can be at least partially attributed to the fact that chelerythrine and sanguinarine are reported to inhibit COX-2 *in vitro* (W. [38, 39]). Apart from inhibiting the PGE_2_ synthesis, the investigated alkaloid fraction decreased the production of TNF*α*. Several studies revealed that both alkaloids inhibit TNF*α* production *in vitro* [27, 40]. The results obtained by Meng et al. allow hypothesizing that the observed decrease of the TNF*α* concentration may be at least partially the consequence of the inhibitory influence of sanguinarine on TLR4/NF*κ*B signalling pathway [8].

An important role in the progress of inflammation is played by zinc-dependent proteolytic enzymes—matrix metalloproteinases (MMP), including MMP-9. In pathophysiological conditions, MMP-9 is upregulated during development and wound healing as well as during pathologies that involve inflammatory processes, including arthritis, diabetes, and cancer [41]. Certain dependence of COX expression on the presence of MMP-9 was also proved [42]. The imbalance between synthesis and degradation of MMP-9 contributes to inadequate tissue remodeling, which can consequently lead to the formation of ulcers in the mucosa [43]. It was shown that MMP-9 is one of the key enzymes involved in the degradation of intestinal tissue during an inflammatory disease of gastrointestinal tract, for example, Crohn's disease (CD) and ulcerative colitis (UC) [44, 45]. In various experimental animal models, it was observed that the decrease of MMP-9 can result in the attenuation of inflammation in the intestine [46, 47]. In the present study, we observed the increased level of MMP-9 in the paw of carrageenan-administered animals. We have shown that the tested alkaloid fraction (as well as the positive control—indomethacin) significantly reduced the concentration of MMP-9 evoked by the inflammation induced by the carrageenan administration. Park et al. (S. Y. [48]) informed that sanguinarine inhibited TPA-induced MMP-9 mRNA and protein expression and MMP-9 enzymatic activity in a dose-dependent manner in the breast cancer model. Their examination also proved sanguinarine to reduce COX-2 and PGE_2_ levels. Thus, the decrease in PGE_2_ secretion reported in our study is in line with the above-mentioned report of Park et al. Depletion of MMP-9 expression in response to sanguinarine [49] and to chelerythrine has also been observed in other studies, where the inactivation of NF*κ*B pathway was concomitantly noted [25, 50, 51]. However, to our knowledge, up to date, no published reports have examined the impact of sanguinarine and chelerythrine on MMP-9 concentration in the classic inflammation model. Therefore, our findings are the first to suggest that this may be one of the mechanisms underlying the anti-inflammatory activity of both alkaloids.

It is worth noting that the anti-inflammatory activity of the *C. chinensis* fraction containing sanguinarine and chelerythrine was in multicriteria decision analysis comparable (groups SC_5_ and SC_10_) to that of indomethacin—a drug considered to be one of the strongest NSAIDs. However, the use of indomethacin in clinical practice is relatively limited, mostly to external use, e.g., in the form of an aerosol, mainly due to its ulcerogenic effect. In fact, indomethacin is commonly used orally for more serious conditions, such as arthritis. Taking into account the results of our study and recently published paper showing the effectiveness of sanguinarine in the treatment of neuropathic pain in animal models (P. [52]), we believe that investigated alkaloids may be a very valuable alternative to indomethacin, as their anti-inflammatory potency is comparable, but practically devoid of the acute ulcerogenic side effect of indomethacin (groups SC_5_ and SC_10_). Obviously, this evaluation should take into account the short duration of the experiment and the single one exposure of the tissue to the inflammatory factor. Due to the fact that indomethacin if applied is most commonly used in chronic inflammatory diseases, therefore, since the results of our study showed a certain therapeutic potential of the investigational fraction, further analyses are necessary for the complete comparison, including assays that would include multiple administration of the SC fraction and evaluation of its effects in the case of chronic exposure to inflammation. Sanguinarine and chelerythrine are characterized by a highly homologous structure; however, they differ in varied oxygen electron-donating substituents, which may potentially result in the diversified intensity of their anti-inflammatory effects [53]. An influential difference was also observed in the case of the anticancer effect. Many cancer cells develop a mechanism to foreclose programmed cell death through the overproduction of proteins that prevent apoptosis, e.g., Bcl-2 and Bcl-XL. Sanguinarine and chelerythrine may inhibit these proteins, thus leading to the death of cancer cells [54, 55]. Despite the structural homology between these two compounds, they appear to bind to various target regions of the Bcl-XL protein, and in both cases, the docking points are different than in other known Bcl-XL inhibitors (Y.-H. [56]). The above results may suggest that there might be a potential additive synergism between these two compounds (due to e.g. various target points or intensity of particular molecular mechanisms), which could also be significant in terms of their anti-inflammatory activity, and the mixture of both alkaloids may be more effective than if substances were used individually. As our examination of the effects of the SC fraction have yielded promising results, further research, including comparison of the anti-inflammatory effects of the mixture and each of the compounds individually, is more than recommended.

In the present study, pretreatment with indomethacin was associated with a significant macroscopic and microscopic damage of gastric mucosa, being the sign of acute gastrotoxicity. However, we did not detect any acute ulcerogenic activity of investigated fraction. Macroscopic and microscopic assessments of the gastric mucosa revealed significant gastric damage in animals receiving indomethacin, whereas the stomachs in animals receiving tested alkaloids remained unaffected. The safer gastric profile of the chelerythrine-sanguinarine fraction suggests that these alkaloids inhibit COX-1 activity to a lesser extent than indomethacin. They may be selective or preferential COX-2 inhibitors, but further researches are needed to explore the actual influence of the investigated fraction of *C. chinensis* on COX-1 and COX-2 activity. Our results are in line with the observations reported by Khayyal et al. [57] that described ulceroprotective effect of Iberogast containing among other alkaloids derived from *C. majus*. The gastroprotective effect of chelerythrine and sanguinarine in an animal model of ethanol-induced gastric ulcer was also reported by other authors (W. [38, 58]). Moreover, these alkaloids not only do not exhibit ulcerogenic effects but can also play even a prophylactic role. One of the most important risk factors for peptic ulcer disease is *Helicobacter pylori* infection. Mahady et al. proved that sanguinarine and chelerythrine can inhibit the growth of the bacteria, with a MIC50 of 50.0 and 100.0 *μ*g/mL, respectively [59].

Interestingly, usage of the assessed fraction of *C. chinensis* did not cause a significant alteration in pH of the gastric juice of the tested animals (groups receiving 5 and 10 mg/kg of investigational alkaloid fraction; only the SC_1_ group showed a relevant increase compared to the IND group). This fact also may be of key importance in the context of the possible application of both compounds in clinical practice. Changes in the pH of gastric juice may have undesirable consequences, among other indigestions, decreased appetite, or dyspeptic disorders. Thus, the three observations made in our study: anti-inflammatory activity of tested alkaloids comparable to indomethacin, no pathological changes in the gastric mucosa, and no increase in gastric juice pH in the SC_5_ and SC_10_ groups, make up a very promising whole, potentially presenting higher doses of the sanguinarine-chelerythrine fraction of *C. chinensis* as an effective and at the same time relatively safe anti-inflammatory agent for therapeutic praxis.

## 5. Conclusion

Inflammatory diseases are a common therapeutic problem and nonsteroidal anti-inflammatory drugs are not deprived of side effects, of which ulcerogenic activity is one of the most frequent. In our study, we found that sanguinarine and chelerythrine fraction of natural origin possesses anti-inflammatory activity comparable to indomethacin, but without acute adverse effects on the gastric mucosa. We showed that these isoquinoline alkaloids isolated in a form of fraction from *C. chinensis* inhibited the second phase of carrageenan rat paw oedema in a dose-dependent manner, suggesting the inhibition of PGE_2_ release, decreased the production of TNF*α*, and reduced the concentration of MMP-9. The obtained results present the fraction of sanguinarine and chelerythrine as a promising candidate for further research on new anti-inflammatory and analgesic drugs characterized with a safer gastric profile compared to existing NSAIDs.

## Figures and Tables

**Figure 1:** Chemical structures of sanguinarine (a) and chelerythrine (b).

**Figure 2:** Paw oedema in the experimental groups. CON: negative control group; CAR: positive control group; IND: group receiving indomethacin 10 mg/kg; SC_1_, SC_5_, and SC_10_ : groups receiving investigational alkaloid fraction of *C. chinensis* containing sanguinarine and chelerythrine (1, 5, and 10 mg/kg, respectively). Data are presented as the mean ± SD. ^∗∗∗∗^*p* < 0.0001*vs.* CON, ^#^*p* < 0.05 and^##^*p* < 0.01*vs.* CAR.

**Figure 3:** Paw oedema in the experimental groups. CON: negative control group; CAR: positive control group; IND: group receiving indomethacin 10 mg/kg; SC_1_, SC_5_, and SC_10_ : groups receiving investigational alkaloid fraction of *C. chinensis* containing sanguinarine and chelerythrine (1, 5, and 10 mg/kg, respectively).

**Figure 4:** Inhibition of the paw oedema with indomethacin and investigational mixture 6 hours after the injection of 1% carrageenan solution. IND: group receiving indomethacin 10 mg/kg; SC_1_, SC_5_, and SC_10_: groups receiving an investigational fraction of *C. chinensis* containing sanguinarine and chelerythrine (1, 5, and 10 mg/kg, respectively). Data are presented as the mean ± SD. ^∗^*p* < 0.05*vs*. IND.

**Figure 5:** Macroscopic examination of the gastric mucosa. Experimental groups (*n* = 10): (a) group receiving investigational alkaloid fraction of *C. chinensis* containing sanguinarine and chelerythrine 1 mg/kg (SC_1_); (b) group receiving investigational alkaloid fraction of *C. chinensis* containing sanguinarine and chelerythrine 5 mg/kg (SC_5_); (c) group receiving investigational alkaloid fraction of *C. chinensis* containing sanguinarine and chelerythrine 10 mg/kg (SC_10_); (d) group receiving indomethacin 10 mg/kg (IND); (e) positive control group (CAR); (f) negative control group (CON).

**Figure 6:** Microscopic examination of the gastric mucosa after hematoxylin-eosin (H&E) staining (×100). Experimental groups (*n* = 10): (a) group receiving investigational alkaloid fraction of *C. chinensis* containing sanguinarine and chelerythrine 1 mg/kg (SC_1_); (b) group receiving investigational alkaloid fraction of *C. chinensis* containing sanguinarine and chelerythrine 5 mg/kg (SC_5_); (c) group receiving investigational alkaloid fraction of *C. chinensis* containing sanguinarine and chelerythrine 10 mg/kg (SC_10_); (d) group receiving indomethacin 10 mg/kg (IND); (e) positive control group (CAR); (f) negative control group (CON). In CAR group (e) and SC_1_ group (a) generally normal mucosa showing a mild inflammation was detected. In indomethacin receiving animals (d) moderate inflammation and ulceration in the mucosa was present. In (b), (c), and (f), normal mucosa with no inflammation was observed.

**Figure 7:** Multicriteria decision analysis (MCDA) of the anti-inflammatory effect of investigational groups. IND: group receiving indomethacin 10 mg/kg; SC_1_, SC_5_, and SC_10_ : groups receiving investigational fraction of *C. chinensis* containing sanguinarine and chelerythrine (1, 5, and 10 mg/kg, respectively). Data are presented as the mean ± SD. ^∗^*p* < 0.05*vs*. IND.

**Table 1:** The influence of the investigational alkaloid fraction of *C. chinensis* containing sanguinarine and chelerythrine on the levels of TNF*α*, PGE_2_, and MMP-9 in the homogenized subplantar tissue.

Group	TNF*α* (pg/mL)	PGE_2_ (pg/mL)	MMP-9 (pg/mL)
CON	18.797 ± 7.793^#^	8.797 ± 2.798^###^	0.020 ±0.049^####^
CAR	61.117 ± 32.457	35.275 ± 19.856	4.360 ± 3.520
IND	25.800 ± 14.629^#^	2.500 ± 0.548^####^	0.000 ± 0.000^####^
SC_1_	22.611 ± 22.357^#^	10.149 ± 6.161^####^	0.000 ± 0.000^####^
SC_5_	10.597 ± 4.530^##^	7.443 ± 7.257^###^	0.000 ± 0.000^####^
SC_10_	24.369 ± 3.799^#^	3.600 ± 2.074^####^	0.000 ± 0.000^####^

TNF*α*: tumour necrosis factor alpha; PGE_2_: prostaglandin E_2_; MMP-9: matrix metalloproteinase 9; CON: negative control group; CAR: positive control group; IND: group receiving indomethacin 10 mg/kg; SC_1_, SC_5_, and SC_10_ : groups receiving an investigational fraction of *C. chinensis* containing sanguinarine and chelerythrine (1, 5, and 10 mg/kg, respectively). Data are presented as the mean ± SD. ^#^*p* < 0.05,  ^##^*p* < 0.01,  ^###^*p* < 0.001, and^####^*p* < 0.0001*vs.* CAR.

**Table 2:** The impact of investigational alkaloid fraction of *C. chinensis* containing sanguinarine and chelerythrine on gastric mucosa. Indomethacin was used as a reference drug.

Group	Macroscopic evaluation	Microscopic evaluation (H&E staining)		
	Gastric index	Inflammation score (0-3)	Gastric mucosa damage score (0-3)	Cumulative microscopic gastric index (0-6)
CON	0.50 ± 0.71^∗∗∗∗^	0.571 ± 0.787^∗∗∗∗^	0.143 ± 0.378^∗∗∗∗^	0.714 ± 1.113^∗∗∗∗^
CAR	0.64 ± 1.08^∗∗∗∗^	0.875 ± 0.354^∗∗∗∗^	0.0 ± 0.0^∗∗∗∗^	0.875 ± 0.354^∗∗∗∗^
IND	17.90 ± 8.56^∧∧∧∧^	1.375 ± 0.518^∧∧∧∧^	1.375 ± 0.518^∧∧∧∧^	2.750 ± 0.886^∧∧∧∧^
SC_1_	0.0 ± 0.0^∗∗∗∗^	0.375 ± 0.518^∗∗∗∗^	0.125 ± 0.354^∗∗∗∗^	0.500 ± 0.756^∗∗∗∗^
SC_5_	0.20 ± 0.42^∗∗∗∗^	0.0 ± 0.0^∗∗∗∗^	0.0 ± 0.0^∗∗∗∗^	0.0 ± 0.0^∗∗∗∗^
SC_10_	0.0 ± 0.0^∗∗∗∗^	0.250 ± 0.463^∗∗∗∗^	0.0 ± 0.0^∗∗∗∗^	0.250 ± 0.463^∗∗∗∗^

CON: negative control group; CAR: positive control group; IND: group receiving indomethacin 10 mg/kg; SC_1_, SC_5_, and SC_10_ : groups receiving investigational alkaloid fraction of *C. chinensis* containing sanguinarine and chelerythrine (1, 5, and 10 mg/kg, respectively); H&E: hematoxylin-eosin. The severity of macroscopic gastric damage was evaluated using the J-scoring method, classifying the erosions as follows: no erosions = 0; 0-1 mm in diameter = 1; 1-2 mm = 2; greater than 2 mm in diameter = 3. The sum of these measured areas in each animal was described as the cumulative macroscopic gastric index [31]. Microscopic evaluation assessed independently the inflammation process and the damage of gastric mucosa. The severity of the inflammation was assessed using 0-3 scale (0: no inflammation, 1: mild inflammation, 2: moderate, and 3: severe inflammation). The severity of the damage of gastric mucosa was assessed using 0-3 scale (0: no damage, 1: superficial erosion, 2: submucous ulceration, and 3: ulceration in muscularis propria). The cumulative microscopic gastric index was defined as the sum of the inflammation and damage score. Data are presented as the mean ± SD. ^∗∗∗∗^*p* < 0.0001*vs.* IND; ^^^^^^*p* < 0.0001*vs.* CON.

**Table 3:** The impact of investigational alkaloid fraction of *C. chinensis* containing sanguinarine and chelerythrine on pH of gastric juice. Indomethacin was used as a reference drug.

Group	pH
CON	3.157 ± 0.457
CAR	3.450 ± 0.761
IND	3.234 ± 0.603
SC_1_	4.282 ± 0.391^##^
SC_5_	3.274 ± 0.368
SC_10_	3.464 ± 0.756

CON: negative control group; CAR: positive control group; IND: group receiving indomethacin 10 mg/kg; SC_1_, SC_5_, and SC_10_ : groups receiving investigational alkaloid fraction of *C. chinensis* containing sanguinarine and chelerythrine (1, 5, and 10 mg/kg, respectively). Data are presented as the mean ± SD. ^##^*p* < 0.01*vs.* IND.

## Data Availability

The data underlying this article will be shared upon request to the corresponding author.
